# Effects of Infrared Combined with Methylcobalamin on the Vibratory Sensory Threshold and Nerve Conduction Velocity of the Lower Extremity in Patients with Diabetic Foot Treatment

This article has been retracted.

**DOI:** 10.1155/2022/8287192

**Published:** 2022-08-28

**Authors:** Yi Wang, Shaona Lin, Zongcun Chen, Qinghua Chen, Maoxiong Fu

**Affiliations:** Department of Endocrinology, The Second Affiliated Hospital of Hainan Medical University, China

## Abstract

**Objective:**

To investigate the effect of infrared combined with methylcobalamin on the vibratory sensory threshold and lower limb nerve conduction velocity of patients with diabetic foot.

**Methods:**

One hundred and six patients with diabetic foot in our hospital from February 2018 to December 2020 were enrolled and divided into the study and control groups. The patients in the control group were given methylcobalamin, and the patients in the research group were treated with infrared light on the basis of the control group. The therapeutic effect, vibration sensory threshold, lower limb nerve conduction velocity, and related biochemical index levels before and after treatment in the two groups were counted.

**Result:**

The total effective rate of the study group (94.34%) was significantly higher than that of the control group (81.13%). The left/right lower limb vibration sensation threshold decreased in both groups after treatment, and the study group was lower than that of the control group (*P* < 0.05). The conduction velocity of the left/right common peroneal nerve and tibial nerve increased in both groups after treatment, and the study group was larger than that of the control group (*P* < 0.05). The bFGF, VEGF, and APN increased in both groups after treatment. VEGF and APN increased and IL-6 and TNF-*α* decreased in both groups after treatment, and the study group was better than the control group (*P* < 0.05).

**Conclusion:**

Infrared and methylcobalamin combined treatment of diabetic foot can effectively improve lower extremity nerve conduction velocity and vibration sensory threshold, regulate serum bFGF and VEGF levels, reduce the degree of inflammatory response, and help improve the overall treatment effect.

## 1. Introduction

Diabetic foot is an important complication of diabetes. In recent years, the incidence of diabetes has been on the rise, and the number of diabetic foot patients has been increasing. Different degrees of vascular disease cause lower extremity pain, ulcers, infection and deep tissue damage [1]. The diabetic foot is prone to recurrence, long duration, and difficult to heal, and patients are prone to poor nutrition due to their excessive consumption, which can lead to amputation in severe cases [2]. The pathogenesis of diabetic foot is complex, not only related to impaired lipid metabolism, insulin resistance, vascular endothelial function damage caused by long-term hyperglycemia, infection, hypercoagulability and abnormal blood rheology but also closely related to microinflammatory response [3]. Methylcobalamin is a common therapeutic drug for diabetic foot, which can repair nerve tissues and promote regeneration of axonal injury but is less effective when applied alone [4]. Infrared therapy also plays an important role in diabetic foot, by irradiating the local wound and increasing its temperature, thereby regulating the microcirculation and metabolic state of the tissue and accelerating wound healing [5]. Based on this, the purpose of this study was to select patients with diabetic foot in our hospital and group them to explore the value of infrared combined with mecobalamin therapy.

## 2. Methods

### 2.1. General Information

One hundred and six patients with diabetic foot in our hospital from February 2018 to December 2020 were selected and divided into the study group and control group based on the random number table method. The protocol of this study was approved by ethical committee of the Second Affiliated Hospital of Hainan Medical University. All patients signed the consent forms.

### 2.2. Selection Criteria

The inclusion criteria were as follows: (1) diagnosis confirmed by clinical examination and physical signs [16], (2) intact foot, (3) age < 80 years, (4) informed consent of the patient or family, and (5) good compliance. The exclusion criteria were as follows: (1) those with acute complications of diabetes, (2) those with cognitive dysfunction and communication impairment, (3) those with hyperosmolar coma and ketoacidosis, and (4) those with aortitis, thrombo-occlusive vasculitis, Raynaud's syndrome, and other vascular lesions.

### 2.3. Methodology

In the control group, mecobalamin was administered intravenously at 0.5 mg + 100 mL of saline, once per day. In the study group, infrared therapy was administered based on the control group, and the KP-220 infrared therapy instrument (Hainan Longteng Medical Equipment Co., Ltd.) was used for treatment, with the lamp head of the instrument placed at about 30-40 cm on the affected limb, and the power was set to 32 mW/cm^2^, with a wavelength of 2-25 *μ*m. Both groups were treated for 4 weeks.

### 2.4. Observed Indicators

(1) The effect of treatment in both groups was counted, and the increase in neuromotor and sensory conduction velocity of >20% was considered effective. The increase in neuromotor and sensory conduction velocity of 10%-20% was considered show effect. The increase in neuromotor and sensory conduction velocity of less than the above criteria was considered ineffective. The ‘show effect' and ‘effective' was counted as the total effective rate. (2) The vibrosensory thresholds of the two groups before and after treatment were measured by the vibrosensory threshold detector (Bio Thesiometer, USA). (3) The nerve conduction velocity of the lower limbs before and after the treatment in the two groups was calculated, and the conduction velocity of the left/right common peroneal nerve and tibial nerve were measured by neuromyography. (4) The levels of biochemical indexes, such as basic fibroblast growth factor (bFGF), vascular endothelial growth factor (VEGF), interleukin-6 (IL-6), tumor necrosis factor-*α* (TNF-*α*), and lipocalin (APN), were determined by ELISA kits (ProteinTech, China) before and after treatment in both groups, and blood samples were drawn and measured by the enzymatic method.

### 2.5. Statistical Analysis

The statistical analysis was performed by using SPSS 22.0 (IBM SPSS Statistics, Chicago, USA). The measurement data were expressed as mean ± *s* and analyzed by *t*-test. The count data were expressed as n (%) and analyzed by Chi-square test. A two-sided *P* value less than 0.05 was considered a statistically significant difference.

## 3. Results

### 3.1. Treatment Effect

There were 29 male and 24 female cases in the study group; age 53-79 years, mean 65.98 ± 12.02 years; disease duration 1-6 years, mean 3.53 ± 1.49 years; and body mass index (BMI) 18.4-27.3 kg/m^2^, mean 22.85 ± 3.39 kg/m^2^. There were 31 male and 22 female cases in the control group; age 52-79 years, mean 66.37 ± 10.95 years old; disease duration 1-8 years, mean 4.02 ± 1.61 years; and BMI 18.1-27.9 kg/m^2^, mean 23.05 ± 3.51 kg/m^2^. Baseline data of the two groups were balanced and comparable (*P* > 0.05). As shown in Table 1, the total effective rate of the study group (94.34%) was significantly higher than that of the control group (81.13%) (*P* < 0.05).

### 3.2. Vibration Sensory Threshold

There was no significant difference between two groups in the left/right lower extremity vibration sensory thresholds before treatment (*P* > 0.05), and the left/right lower extremity vibration sensory thresholds decreased in both groups after treatment, and the study group was significantly lower than the control group (*P* < 0.05, Table 2).

### 3.3. Lower Limb Nerve Conduction Velocity

Before treatment, there were no significant differences in conduction velocity of the left/right common peroneal nerve and tibial nerve between two groups (*P* > 0.05). After treatment, the study group was significantly higher than the control group (*P* < 0.05, Table 3).

### 3.4. Biochemical Indicators

There was no significant difference between bFGF, VEGF, IL-6, TNF-*α*, and APN in the two groups before treatment (*P* > 0.05). bFGF, VEGF, and APN increased and IL-6 and TNF-*α* decreased in the two groups after treatment, and the study group was significantly higher than the control group (*P* < 0.05, Table 4).

## 4. Discussion

The development of diabetic foot is mainly due to the long-term high level of blood glucose, which leads to a decrease in the oxygen-carrying capacity of red blood cells and an increase in blood viscosity, making it easy for local blood supply, vascular inflammatory reaction, vascular sclerosis, etc., and can cause autonomic, sensory and motor neuropathy, and eventually diabetic foot [6, 7]. At the same time, if the diabetic foot does not receive timely and effective intervention, it may lead to many complications and even require amputation, so timely treatment of patients is essential [8].

Methylcobalamin is a commonly used drug for the treatment of diabetic foot. It is a methylated vitamin B_12_, which is widely distributed in peripheral nerves and can be transported to nerve cells to stimulate the synthesis of lecithin and axonal pulp proteins by transmethylation, repair myelin, and accelerate the regeneration of damaged axons, thus regulating nerve conduction speed and relieving patients' symptoms [9]. It has also been pointed out that mecobalamin is an endogenous B_12_, which can participate in the carbon unit cycle and has an important role in the homocysteine synthesis protein acid transmethylation reaction, and is extremely suitable for lower limb neuropathy [10]. Meanwhile, methylcobalamin has strong affinity for nerves, which can promote nerve regeneration and increase the blood flow in the nerve endothelium, regulate the neurotrophic state, and enhance the conduction speed of motor nerves [11]. Infrared therapy instrument is an important physical therapy for diabetic foot, which can irradiate deep tissues by combining infrared and red light, and the heat generated during infrared therapy can stimulate local blood vessels by acting on damaged parts, which can effectively dilate, improve local blood circulation, reduce nerve tissue hypoxia and ischemia, and restore local tissue oxygen and nutrient supply, thus shortening the healing time of the wound [12, 13]. The results of this study showed that the total efficiency of the study group was higher than that of the control group, and the vibratory sensory threshold and nerve conduction speed of the lower limbs were better than those of the control group (*P* < 0.05), which confirmed that the combined treatment of diabetic foot with methylcobalamin and infrared rays could effectively regulate the state of the lower limbs and facilitate the improvement of the treatment effect of the disease. After the heat stimulates the nerve reflexes of the body, it can dilate the blood vessels in the body, accelerate the local blood flow, and ensure the nutrient supply to the limbs [14]. Robinson et al. [15] also pointed out that infrared therapy has strong penetration and low quantum energy and does not burn the body, and the local irradiation can convert the infrared energy absorbed by the skin and subcutaneous tissues into heat energy, which can induce the endothelial cells of blood vessels to produce nitric oxide, thus triggering the vasodilation of blood vessels, accelerating blood flow, and restoring the disease. The local irradiation can convert the infrared energy absorbed by the skin and subcutaneous tissues into heat energy, prompting the endothelial cells of blood vessels to produce nitric oxide, thus triggering the expansion of blood vessels, accelerating blood flow, restoring local microcirculation and nutrient supply, achieving the goal of anti-infection, and promoting wound healing.

VEGF is a proangiogenic factor with central mediating function, which can promote the proliferation and division of endothelial cells and accelerate the formation of new blood vessels. In this study, the levels of bFGF and VEGF in the study group were higher than those in the control group after treatment (*P* < 0.05), suggesting that mecobalamin combined with infrared therapy can promote angiogenesis and thus ensure good wound healing. In addition, IL-6 and TNF-*α* are inflammatory factors and their serum expression are positively correlated with the inflammatory response in vivo, while APN is a specific type of protein for adipocyte production and has functions such as regulating glucolipid metabolism, which can regulate the inflammatory response of vascular endothelial cells. In this study, the levels of IL-6, TNF-*α*, and APN in the study group were better than those in the control group after treatment (*P* < 0.05), which further confirmed the high value of the combined intervention program of methylcobalamin and infrared light, which can regulate the degree of inflammatory response in vivo and help to ensure good disease regression.

In conclusion, the combination of infrared light and methylcobalamin in the treatment of diabetic foot can effectively improve the nerve conduction velocity and vibratory sensory threshold of the lower extremity, regulate the serum bFGF and VEGF levels, reduce the degree of inflammatory response, and contribute to the overall treatment effect.

## Figures and Tables

**Table 1:** Comparison of treatment effects between the two groups.

Group	Number of cases	Show effect	Effective	Invalid	Total efficiency
Research group	53	29 (54.72%)	21 (39.62%)	3 (5.66%)	50 (94.34%)
Control group	53	24 (45.28%)	19 (35.85%)	10 (18.87%)	43 (81.13%)
*χ* ^2^ value					4.296
*P* value					0.038

**Table 2:** Comparison of vibration sensation thresholds between the two groups (*V*).

Time	Group	Number of cases	Left side	Right side
Before treatment	Research group	53	20.52 ± 3.49	20.48 ± 4.01
	Control group	53	21.08 ± 3.72	21.11 ± 3.56
	*t* value		0.799	0.855
	*P* value		0.426	0.394

After treatment	Research group	53	14.98 ± 2.96	15.40 ± 2.53
	Control group	53	17.42 ± 2.85	17.71 ± 2.54
	*t* value		4.323	4.691
	*P* value		<0.001	<0.001

**Table 3:** Comparison of lower limb nerve conduction velocities between the two groups (m/s).

Time	Group	Number of cases	Common peroneal nerve		Tibial nerve	
			Left side	Right side	Left side	Right side
Before treatment	Research group	53	41.23 ± 3.58	34.29 ± 5.51	43.50 ± 3.57	43.96 ± 2.87
	Control group	53	40.08 ± 3.97	33.67 ± 5.45	44.12 ± 4.13	44.56 ± 3.21
	*t* value		1.566	0.582	0.827	1.014
	*P* value		0.120	0.562	0.410	0.313

After treatment	Research group	53	50.02 ± 4.04	44.23 ± 5.12	51.22 ± 2.85	51.79 ± 3.37
	Control group	53	45.37 ± 3.44	39.99 ± 4.55	48.54 ± 3.23	46.71 ± 3.18
	*t* value		6.380	4.506	4.529	7.982
	*P* value		<0.001	<0.001	<0.001	<0.001

**Table 4:** Comparison of biochemical indicators between the two groups.

Time	Group	Number of cases	VEGF (ng/L)	bFGF (ug/L)	IL-6 (pg/mL)	TNF-*α* (ng/mL)	APN (ug/L)
Before treatment	Research group	53	102.18 ± 11.45	25.79 ± 5.54	321.24 ± 21.18	3.89 ± 0.72	16.58 ± 3.45
	Control group	53	100.78 ± 13.85	26.08 ± 6.24	318.30 ± 25.64	4.01 ± 0.69	17.14 ± 3.88
	*t* value		0.567	0.253	0.644	0.876	0.785
	*P* value		0.572	0.801	0.521	0.383	0.434

After treatment	Research group	53	141.23 ± 15.15	40.68 ± 6.43	189.02 ± 19.45	2.69 ± 0.48	26.60 ± 3.67
	Control group	53	122.68 ± 13.64	35.14 ± 5.82	242.11 ± 23.45	3.39 ± 0.51	21.78 ± 3.04
	*t* value		6.625	4.650	12.686	7.276	7.363
	*P* value		<0.001	<0.001	<0.001	<0.001	<0.001

## Data Availability

The authors confirm that the data supporting the findings of this study are available within the article.
